The article "Diagnostic Value of Color Doppler Ultrasonography in Subacute Thyroiditis" was retracted in 2023. Reasons: signs of a paper mill; compromised peer review; unreliable results or conclusions.

# Diagnostic Value of Color Doppler Ultrasonography in Subacute Thyroiditis

**DOI:** 10.1155/2022/7456622

**Published:** 2022-09-17

**Authors:** Yonggang Chen, Shulan Zhu, Huabin Chen, Liting Yao, Jingmian Zhou, Yi Xu, Biqin Lin, Xiaoping Chen

**Affiliations:** ^1^Department of Ultrasound, Fujian Medical University Xiamen Humanity Hospital, Xiamen, Fujian 361006, China; ^2^Department of Ultrasound, Zhongshan Hospital of Xiamen University, School of Medicine, Xiamen University, Xiamen, Fujian 361004, China; ^3^National Demonstration Center for Experimental Electronic Information Education, Xiamen University, Xiamen, Fujian 361004, China

## Abstract

In order to explore the clinical effect of color Doppler ultrasonography in the diagnosis of subacute thyroiditis, a method for the diagnosis of subacute thyroiditis by color Doppler ultrasonography was proposed. From November 2019 to November 2020, 90 patients with subacute thyroiditis in our hospital were selected as the experimental group; 90 healthy people were selected as the control group during the same period. Both groups were diagnosed by color Doppler ultrasonography and compared. The experimental results showed that patients with subacute thyroiditis showed mild to moderate enlargement of the involved thyroid gland, and local or diffuse inhomogeneous hypoechoic areas may appear in bilateral or unilateral thyroid glands: irregular edges, unclear boundaries, no “ball feel,” mottled changes, and accompanied by tenderness. The blood flow signal around the hypoechoic area is rich, and the internal blood flow signal is less. There was no significant increase in the blood flow velocity of the superior thyroid artery on the affected side. Color Doppler ultrasound not only is simple, economical, and non-invasive but also has a good diagnostic accuracy for subacute thyroiditis, which can provide an important basis for clinical diagnosis and treatment and is worthy of popularization and application.

## 1. Introduction

Thyroiditis is a series of clinical symptoms caused by pathological changes of thyroid tissue such as degeneration, exudation, necrosis, and hyperplasia. Among them, the incidence rate of Hashimoto's thyroiditis and subacute thyroiditis is relatively high. The course of thyroiditis is dynamic, which can be characterized by normal thyroid function, transient hyperthyroidism, or hypothyroidism, and a few patients will develop into permanent hypothyroidism [1]. The ultrasonic manifestations of thyroiditis in different stages will also be different. According to the different manifestations of ultrasonography, thyroiditis can be divided into diffuse type, focal type, and nodular type. Focal thyroiditis may be an early manifestation of thyroiditis or a chronic manifestation of thyroiditis. Compared with diffuse thyroiditis, it can be characterized by single or multiple nodular echoes on ultrasound. When the background of thyroid parenchyma is relatively normal, its sonogram can be diverse, which has many similarities with thyroid microcarcinoma. Subacute thyroiditis (SAT) is a common clinical thyroiditis. It is generally believed that SAT may be caused by thyroid injury caused by viral infection, and autoimmune response also plays a role in the occurrence and development of the disease. Subacute thyroiditis is a common clinical disease. There are many factors inducing the disease, and the condition is relatively complex. The health level of patients with the disease will decline, which will have a certain impact on their normal life. In the early stage of subacute thyroiditis, the disease starts rapidly, and patients often have chills, fear of cold, loss of appetite, fatigue, and weakness. If they do not see a doctor in time, the disease is easy to develop, leading to more serious diseases. Therefore, it is very important to choose a scientific, reasonable, and accurate diagnostic method in clinic. Color Doppler ultrasound diagnosis is a common clinical diagnosis method. In recent years, with the continuous development of medical technology, color Doppler ultrasound diagnosis technology is also improving. In the diagnosis of subacute thyroiditis, color Doppler ultrasound can better observe the thyroid condition of patients, so as to diagnose the disease. The color ultrasound diagnostic images of patients with subacute thyroiditis are generally diffuse. After the focus of thyroiditis, there will be enlargement of one lobe and uneven echo. At the same time, when observing the patient's thyroid sonogram, there may also be single or multiple irregular hypoechoic areas. These echo areas have no clear boundary and contour, and the internal echo will also be uneven. The center to the periphery of the sonogram will gradually increase. Some patients will also have no echo due to physiological structure and other factors. In addition, the blood flow signal in the thyroid tissue of patients with subacute thyroiditis is usually not obvious in the low echo area, while the peripheral blood flow signal is gradually enriched, which can show star dot, ring, etc., when the blood vessels in the focus are compressed, the peak velocity of pulse Doppler will also increase. Therefore, the peak systolic velocity of human superior thyroid artery will increase to a certain extent in the presence of subacute thyroiditis. There is no obvious blood flow change in normal thyroid tissue, and there will be no blood flow signal or pressure bending. Therefore, in the diagnosis of subacute thyroiditis, color Doppler ultrasound diagnosis has significant clinical application value and is widely welcomed by doctors and patients [2].

The article "Diagnostic Value of Color Doppler Ultrasonography in Subacute Thyroiditis" was retracted in 2023. Reasons: signs of a paper mill; compromised peer review; unreliable results or conclusions.

With the clinical application and development of high-frequency ultrasound probe (Figure 1), it can clearly display the image characteristics of nodules with diameter less than 1.0 cm, which has become the first choice for thyroid diseases. The two-dimensional image can show the location, size, range, boundary, and internal echo of thyroid lesions. Combined with color Doppler ultrasound, important information such as blood flow distribution and blood flow velocity of thyroid parenchyma and lesions can be observed. Because the conventional ultrasound manifestations of focal thyroiditis and thyroid micropapillary carcinoma are very similar and the diagnosis is difficult, this paper reviews the color Doppler ultrasound manifestations of 90 patients with subacute thyroiditis, in order to further explore the value of color Doppler ultrasound in the diagnosis and differential diagnosis of subacute thyroiditis [3].

## 2. Literature Review

At present, scholars at home and abroad have done a lot of research on diffuse thyroid diseases such as SAT by using the ultrasonic elastography rating method: Villalba, Landry, and Brown believe that the diagnosis of typical SAT is not difficult. It usually occurs in winter and spring, with acute onset. At the initial stage of onset, it is characterized by pharyngeal pain, fatigue, general discomfort, fever of different degrees, and other symptoms of upper respiratory tract infection, including hoarseness and dysphagia. Thyroid mass and local pain are characteristic clinical manifestations [4]. Amaniampong et al. believe that SAT is multiple and has a good prognosis. Patients with mild symptoms do not need special treatment, can rest properly, and give non glucocorticoid anti-inflammatory and analgesic drugs. Patients with severe systemic symptoms, persistent high fever, goiter, and obvious tenderness can be treated with glucocorticoid. The main purpose of treatment is to reduce symptoms and prevent recurrence [5]. Hu et al. reported that normal thyroid parenchyma is composed of a large number of follicular cells filled with colloid. There are abundant capillaries between the follicles, so the hardness is small. The elastic diagram is mainly green and uniform [1]. Qi et al. reported that in the early stage of SAT, the pathological characteristics are a large number of inflammatory cells infiltrating in the thyroid stroma, destruction of follicles, formation of micro abscess, colloid overflow from microfollicles, surrounded by surrounding tissue cells, and multinuclear giant cells to form granuloma. These changes increase the number of cells per unit volume. In addition to tissue edema caused by inflammatory reaction, the hardness of the focus area will inevitably increase significantly. The elastic rendering of the focus is mainly blue. The research results of this group are also consistent with the literature report [6]. Ichou, Gauvin, and Faingold reported 2 cases of SAT diagnosed by puncture, of which 1 case showed only a small abnormal echo area on conventional ultrasound, but ultrasonic elastic imaging has obviously shown the increase of the hardness of the echo area. These studies suggest that SAT elastogram can display the lesion areas that cannot be displayed in two-dimensional ultrasound, which is of positive significance for accurately evaluating the lesion scope of SAT and finding potential lesions. This study shows that two-dimensional ultrasound was combined with ultrasound elastography [7]. Hua, Wang, and Zhang studied the clinical characteristics of 852 SAT patients before treatment and found that most of the laboratory test results were related to thyrotoxicosis and inflammation and liver dysfunction, and the abnormal peak level often appeared one week after the onset. The whole disease stage of typical SAT patients can be divided into three stages: acute stage with hyperthyroidism, remission stage with hypothyroidism (divided into transition stage and hypothyroidism stage), and recovery stage (normal thyroid function stage) [8]. Moreover, Svedin, Dillon, and Parker have found that when the volume of the lesion is too large and all the ROI contains the lesion tissue, but not the normal tissue for comparison, it is often difficult to obtain a satisfactory ultrasonic elastic image, and the results cannot reflect the real hardness of the lesion. Therefore, this study also introduces the SWV value measured by the ARFI elastic imaging vtq technology as a more objective quantitative index to judge SAT, ARFI compression, and transverse vibration. The transverse vibration propagates to the periphery in the form of shear wave. Vtq technology makes the tissue produce longitudinal. SWV can be calculated by using the time difference and wavelength of adjacent peaks of shear wave, which can be used to reflect the hardness of tissue [9]. Tyurina et al. showed that the elastic strain rate ratio of the best diagnostic effect of benign and malignant thyroid nodules ranged from 2.96 to 4.22. The critical point of SR value in this study was 2.29, which was significantly lower than that in the above study. The reason was related to the small lesions in the malignant group. The change of microlesion hardness cannot be reflected on the elastic image, and the false negative result of elastic imaging is obtained [10].

The article "Diagnostic Value of Color Doppler Ultrasonography in Subacute Thyroiditis" was retracted in 2023. Reasons: signs of a paper mill; compromised peer review; unreliable results or conclusions.

## 3. Experimental Analysis

### 3.1. Subjects

From November 2019 to November 2020, 90 patients with subacute thyroiditis in our hospital were selected as the experimental group. The ratio of male to female patients was 47 : 43. The highest age of the patients was 69 years old, and the lowest was 21 years old, with an average of (40.37 ± 4.36) years old; the longest course of disease was 8 months and the shortest was 3 days, with an average of (45.38 ± 7.25) days [11]. In the same period, 90 healthy persons were selected as the control group, of which the male to female ratio was 55 : 45. The highest age of the patients was 68 years old, and the lowest was 22 years old, with an average of (41.31 ± 3.34) years old. Comparing the clinical data of the two groups, there was no significant statistical significance (*P* > 0.05), and the data were highly comparable [12].

Inclusion criteria: (1) The experimental group was confirmed as subacute thyroiditis by pathological diagnosis. (2) Before this study, the medical staff informed the subjects about the study and obtained the informed consent of the subjects. (3) All subjects were adults. Exclusion criteria: (1) Incomplete clinical data. (2) Combined with other serious diseases. (3) There are contraindications for color Doppler ultrasound diagnosis [13].

### 3.2. Experimental Method

Both groups were diagnosed by color Doppler ultrasound. The first experimental method is instrument selection. In this study, the color Doppler ultrasound diagnostic instrument with the model of LOGIQ E9 and its supporting related equipment are selected, and the probe is set as a wide range imaging linear array with the frequency of 7~14 MHz. The second method is position selection. All subjects shall be in a supine position. During the examination, a pillow shall be placed on the back shoulder of the subject, and the patient is required to stretch his neck and tilt back as much as possible to expose the thyroid area as much as possible [14]. The third method is scan diagnosis. The color Doppler ultrasound diagnostic instrument is used to scan the thyroid region of the subject in multiple sections; fully observe the shape, size, blood flow shape, capsule, and internal echo of the subject's thyroid; and measure the left and right diameter, anterior and posterior diameter, and long diameter of the thyroid, so as to fully understand the condition of the focus. At the same time, properly pressurize the probe, observe whether the subject has tenderness, and then focus on the acoustic image and blood flow characteristics of the focus, so as to further diagnose the disease. The ultrasonic images of all subjects were handed over to professionals for judgment, and the diagnostic results of the two groups were compared [15].

The article "Diagnostic Value of Color Doppler Ultrasonography in Subacute Thyroiditis" was retracted in 2023. Reasons: signs of a paper mill; compromised peer review; unreliable results or conclusions.

### 3.3. Observation Indicators

In this study, the anterior posterior diameter, left and right diameter, and blood flow characteristics of the thyroid gland in the affected and healthy sides of the two groups were used as observation indexes. Among them, the blood flow characteristics include the peak systolic velocity of the affected side superior thyroid artery and the peak systolic velocity of the healthy side superior thyroid artery.

### 3.4. Statistical Analysis

The final data of this study were processed by the spss22.0 data software. The measurement data such as the anterior posterior diameter, left and right diameter of the thyroid gland on the affected side and the healthy side, the peak systolic velocity of the superior thyroid artery on the affected side, and the peak systolic velocity of the superior thyroid artery on the healthy side were expressed by standard deviation (*x* ± *s*). A *t*-test was used, and *P* < 0.05 indicated a statistically significant difference [16].

### 3.5. Experimental Analysis

The anterior and posterior diameters and left and right diameters of the affected lateral lobe thyroid in patients with subacute thyroiditis were significantly larger than those in healthy subjects, *t* = 21.53, 23.57, *P* = 0.001; the difference was statistically significant. There was no significant difference in the anterior and posterior diameter and left and right diameter of thyroid between the two groups, *t* = 0.08 and 0.04, *P* = 0.97 and 0.94. The difference was not statistically significant, as shown in Table 1.

The peak systolic velocity of superior lateral lobe artery in patients with subacute thyroiditis was significantly higher than that in healthy subjects, *t* = 19.72, *P* = 0.001. The difference was statistically significant [2]. There was no significant difference in systolic peak velocity between the two groups, *t* = 1.85, *P* = 0.07; the difference is statistically significant (see Table 2).

In the elastic group, there were 45 lesions, 43 were cured and 2 recurred. The cure rate was 95.6%, and the recurrence rate was 4.4%. In the clinical group, there were 40 lesions, 31 were cured and 9 recurred [3]. The cure rate was 77.5%, and the recurrence rate was 22.5%. There was significant difference between the two groups (*P* < 0.05) (see Table 3).

The area of lesions revealed by two-dimensional ultrasound ranged from 0.42 to 4.20 cm^2^, with an average area of 1.35 + 0.90 cm^2^. The lesion area shown by elastogram ranged from 0.49 to 4.57 cm^2^, with an average area of 1.77 + 0.91 cm^2^. The lesion area shown by elastogram was larger than that shown by two-dimensional ultrasound [4], and the difference was statistically significant (*t* = 2.29, *P* < 0.05) (see Table 4).

The article "Diagnostic Value of Color Doppler Ultrasonography in Subacute Thyroiditis" was retracted in 2023. Reasons: signs of a paper mill; compromised peer review; unreliable results or conclusions.

Compared with the pathological results, the SR of focal thyroiditis was 0.54–7.09, with an average of 1.760.92, and that of thyroid microcarcinoma was 1.21–9.84, with an average of 3.14 + 1.87. The SR of thyroid microcarcinoma was significantly higher than that of focal thyroiditis. There was a significant difference between them by *t*-test (*P* < 0.01). The ROC curve is constructed with sensitivity as the ordinate and 1-specificity as the abscissa, as shown in Figure 2.

## 4. Discussion

Subacute thyroiditis is an autoimmune disease caused by viral infection. Patients often have a history of respiratory tract infection before onset. In the early stage of clinical onset, they often have pharyngeal pain, fever, and upper respiratory symptoms, which can be accompanied by increased erythrocyte sedimentation rate and abnormal thyroid function. The destruction and edema of thyroid follicles can lead to the increase of thyroid volume. The two-dimensional ultrasound image shows flake hypoechoic area, and some of them show nodular changes. Color Doppler ultrasound shows that the blood supply in the hypoechoic area is less than that in the normal tissue, and the blood supply around the nodular type is more abundant. This disease should be differentiated from the following diseases: (1) it should be differentiated from thyroid papillary carcinoma. Most of the lesions in the latter have clear boundaries and internal gravel calcification. Color Doppler flow imaging (CDFI): the blood flow in the lesions is rich. (2) Compared with chronic lymphocytic thyroiditis, the sonogram of the latter showed increased uniformity, obvious isthmus thickening, and CDFI: rich blood flow signals, mostly manifested as “Fire Sea sign.”. (3) Compared with acute suppurative thyroiditis, the latter has a history of severe blood circulation infection such as hyperthermia and sepsis, and ultrasound showed irregular dark areas in the focus area. Two-dimensional ultrasound and color Doppler ultrasound can well show the focus and blood supply of subacute thyroiditis, with characteristic sonographic changes. Combined with clinical manifestations, ultrasound has high diagnostic accuracy and important diagnostic value for subacute thyroiditis.

Thyroiditis is not uncommon in clinic. Most patients are easy to diagnose because of their typical clinical manifestations, such as low fever, anterior cervical pain, goiter, and significantly accelerated ESR. However, some patients still have atypical symptoms in the initial stage of onset, which is difficult to distinguish from diseases such as upper respiratory tract infection, pharyngitis, thyroid nodule, or parenchymal hemorrhage [5]. The results show that the ultrasonic manifestations of subacute thyroiditis have certain characteristics: uneven echo reduction changes in varying degrees appear in the thyroid of all patients, most of which are one or more blurred echo reduction areas (limited type) in unilateral or bilateral thyroid, and a few are diffuse echo reduction changes (diffuse type) in unilateral or bilateral thyroid. There was significant tenderness in all hypoechoic sites, and the thickness of thyroid on the changed side of hypoechoic was significantly higher than that of normal (*P* < 0.01). The above results are consistent with the literature reports. The reason may be related to thyroid follicular destruction, inflammatory cell infiltration, and interstitial edema caused by inflammatory reaction. The more severe the inflammatory reaction is, the more obvious the echo reduction is. Some areas even show “cyst like” changes, but there is no later enhancement effect, so it can be distinguished from the real cystic lesions. In this paper, color ultrasound shows that the blood flow signal in the lesion is generally slightly higher than that in the surrounding normal tissues, but the distribution is uneven. Among them, the blood flow signal distribution in the area with significantly reduced echo is less. This study suggests that the part with more blood flow signal distribution may be the lesion in the early recovery state, while the area with significantly reduced echo has less blood flow distribution due to heavy inflammatory reaction and obvious interstitial edema. Doppler measurement shows that the arterial blood flow in the lesion is characterized by low resistance and low speed [17]. At the same time, although some patients will have increased thyroid hormone levels in the blood in the early stage of the disease, the increase is mild, which is reflected in the limited echo reduction type, and the speed of the superior thyroid artery on the lesion side is not significantly higher than that of normal. In diffuse hypoechoic type, the velocity of superior thyroid artery may be higher than normal due to the large range of lesions and severe condition. In differential diagnosis, diffuse hypoechoic subtype of thyroiditis is similar to Graves' disease and Hashimoto's disease on sonogram, while limited hypoechoic type should be distinguished from papillary thyroid carcinoma and limited Hashimoto's disease. According to the author's experience, the vast majority of subacute thyroiditis show obvious tenderness during pressure scanning of its echo reduction area. This feature is rare in the above other thyroid diseases [18]. If combined with clinical manifestations at the same time, there is generally no great difficulty in differential diagnosis. For a small number of patients with atypical ultrasonic and clinical manifestations, ultrasound-guided puncture biopsy is needed for definite diagnosis.

100 patients were followed up by ultrasound after 1 ~ 6 months of treatment. Among them, 90 cases of hypoechoic areas completely disappeared or significantly narrowed, and 10 cases showed the increase of lesion scope or the change of “wandering shape” of lesions. After increasing the dosage or prolonging the medication time, the lesion areas significantly decreased or disappeared. The above results show that ultrasound can clearly distinguish the clinical treatment effect of subacute thyroiditis. Some authors reported that although most of the hypoechoic areas of subacute thyroiditis disappeared completely after treatment, a small number of patients still had small pieces of slightly hypoechoic areas in their thyroid after long-term follow-up. Two cases were also seen in this paper (after 6 months of observation), but the distribution of blood flow signals in them was close to the surrounding normal thyroid tissue [10]. To sum up, the 2D and CDI manifestations of thyroiditis have certain characteristics, which can not only help the clinical diagnosis and differential diagnosis of the disease but also provide great help for the clinic in judging the treatment effect.

The article "Diagnostic Value of Color Doppler Ultrasonography in Subacute Thyroiditis" was retracted in 2023. Reasons: signs of a paper mill; compromised peer review; unreliable results or conclusions.

## 5. Conclusion

The thyroid lesions in the acute stage of SAT showed the internal punctate or abundant punctate blood flow distribution of the lesions, which was more concentrated without surrounding blood flow. Although the blood flow display distribution was not characteristic, it was different from the blood flow distribution around the lesions of adenoma and nodular goiter. The blood flow distribution of the focus in the acute phase of SAT reflects the inflammatory changes and blood flow changes of the focus in the acute phase. Observing the blood flow of the focus can better reflect the healing process and is a good index to guide the treatment. Two-dimensional ultrasound can show thyroiditis lesions in the acute stage of SAT, which has characteristic ultrasound images. Combined with clinical data, two-dimensional ultrasound has high diagnostic value in the acute stage of SAT. In conclusion, color Doppler ultrasound diagnosis in the diagnosis of subacute thyroiditis can better diagnose the disease and provide more reference data for follow-up treatment. It has high accuracy and safety and is worthy of clinical application.

The article "Diagnostic Value of Color Doppler Ultrasonography in Subacute Thyroiditis" was retracted in 2023. Reasons: signs of a paper mill; compromised peer review; unreliable results or conclusions.

Ultrasound can detect small lesions in the thyroid and can also vividly describe the blood supply and hemodynamic parameters inside and around the lesions. The purpose of applying combined ultrasound technology is to make a more accurate judgment on the nature of thyroid lesions through comprehensive analysis of multiple ultrasound indicators, so as to reduce unnecessary surgery, provide more accurate preoperative diagnosis for patients with thyroid cancer, and guide clinicians to develop more reasonable surgical methods for patients. In recent years, various new ultrasonic technologies have developed rapidly, such as ultrasonic elastic imaging technology, contrast-enhanced ultrasound, ultrasonic firefly technology, and two-dimensional ultrasonic imaging technology, which are constantly widely used in clinic. Interventional ultrasound technology will also develop safer and more advanced in the future, so as to improve the accuracy of puncture. With the further improvement and deepening of ultrasound technology research, ultrasound will have a broader application prospect in the diagnosis and characterization of small thyroid lesions.

## Figures and Tables

**Figure 1:** High-frequency color Doppler ultrasound diagnosis.

**Figure 2:** ROC curve of differential diagnosis between focal thyroiditis and thyroid microcarcinoma by elastic strain rate ratio method.

**Table 1:** Comparison of the anterior and posterior diameters and left and right diameters of thyroid gland in the affected and healthy sides of the two groups.

Group	Number of lateral leaves	Anterior posterior diameter of thyroid	Left and right thyroid diameter
Bilateral lobes in the control group	200	15.12 ± 1.76	21.13 ± 1.74
Experimental group affected lateral lobe	100	20.12 ± 2.17	26.11 ± 2.24
Contralateral lobe of experimental group	100	15.18 ± 1.78	20.23 ± 1.71
*t* (ratio of the affected side of the experimental group to the control group)		22.53	21.57
*P* (ratio of the affected side of the experimental group to the control group)		0.001	0.001
*T* (ratio of healthy side of experimental group to control group)		0.08	0.04
*P* (ratio of healthy side of experimental group to control group)		0.97	0.94

**Table 2:** Comparison of the peak systolic velocity of superior lobar artery on the affected side and healthy side between the two groups.

Group	Number of lateral leaves	Peak systolic velocity of superior artery
Bilateral lobes in the control group	200	22.44 ± 5.24
Experimental group affected lateral lobe	100	35.32 ± 5.33
Contralateral lobe of experimental group	100	21.71 ± 4.24
*t* (ratio of the affected side of the experimental group to the control group)		18.72
*P* (ratio of the affected side of the experimental group to the control group)		0.001
*T* (ratio of healthy side of experimental group to control group)		1.84
*P* (ratio of healthy side of experimental group to control group)		0.07

The article "Diagnostic Value of Color Doppler Ultrasonography in Subacute Thyroiditis" was retracted in 2023. Reasons: signs of a paper mill; compromised peer review; unreliable results or conclusions.

**Table 3:** Comparison of curative effect and course of treatment between the two groups.

Group	Number of lesions/piece	Course of treatment/*D*	Cure rate (%)	Recurrence rate (%)
Elastic group	45	93 ± 18	95.6	4.4
Clinical group	40	85 ± 21	77.5	22.5

**Table 4:** Comparison of elastogram grades between subacute thyroiditis disease group and healthy control group.

Elastic grading	SAT group	Control group	/*P* value
1	0	0	117.48 *P* < 0.01
I	0	31	
II	2	9	
III	55	0	
IV	28	0	

## Data Availability

The data used to support the findings of this study are available from the corresponding author upon request.
